# Impact of workplace bullying and burnout on job satisfaction among Bangladeshi nurses: A cross-sectional study

**DOI:** 10.1016/j.heliyon.2023.e13162

**Published:** 2023-01-24

**Authors:** Saifur Rahman Chowdhury, Humayun Kabir, Nahida Akter, Mohammad Azmain Iktidar, Anjan Kumar Roy, Mahfuzur Rahman Chowdhury, Ahmed Hossain

**Affiliations:** a Department of Public Health, North South University, Dhaka 1229, Bangladesh; b Department of Health Research Methods, Evidence, and Impact, McMaster University, 1280 Main Street West, Hamilton, L8S 4L8, Ontario, Canada; c Grameen Caledonian College of Nursing, Dhaka 1216, Bangladesh; d Penn State Ross and Carol Nese College of Nursing, Penn State University, University Park, PA 16802, USA; e Department of Nursing and Health Science, Jashore University of Science and Technology, Jashore, Bangladesh; f Department of English, North East University Bangladesh, Sylhet 3100, Bangladesh; g Health Services Administration, College of Health Sciences, University of Sharjah, Sharjah, United Arab Emirates

**Keywords:** Job satisfaction, Workplace, Bullying, Burnout, Nurses, Healthcare workers, Healthcare professionals

## Abstract

**Background:**

Job satisfaction is one of the most important but least researched issues in the nursing profession in Bangladesh. This study aimed to investigate how workplace bullying and burnout are related to job satisfaction, as well as determine the factors that are associated with job satisfaction among Bangladeshi nurses.

**Methods:**

Data were collected from Bangladeshi registered nurses between February 26, 2021, and July 10, 2021, in this cross-sectional study. Bullying, burnout, and job satisfaction were measured with the Short Negative Acts Questionnaire [S-NAQ], the Burnout Measure-Short version (BMS), and the Short Index of Job Satisfaction (SIJS-5), respectively. The correlations between age, bullying, burnout, and job satisfaction were assessed using a Pearson's correlation test. In order to investigate the adjusted association of demographic characteristics, occupational variables, bullying, and burnout with job satisfaction, multiple linear regression models were fitted.

**Results:**

The study included 1,264 nurses (70.02% were female) with a mean age of 28.41 (±5.54) years. Job satisfaction was significantly negatively correlated with bullying and burnout (p < 0.001). According to the multiple linear regression models, the private-employed nurses had lower job satisfaction than the government-employed nurses (β = −0.901, CI: −1.640 to −0.162). Compared to the nurses in the Dhaka division, the nurses in the Chattogram division (β = 0.854, CI: 0.099 to 1.609) and other divisions (β = 0.993, CI: 0.273 to 1.713) had higher job satisfaction. Nurses without sufficient equipment to manage patients (β = −1.230, CI: −1.696 to −0.763), and nurses not paid on time (β = −1.475, CI: −2.221 to −0.729) were predicted to have significantly lower job satisfaction. Nurses’ job satisfaction levels were decreased with higher levels of workplace bullying (β = −0.086, CI: −0.120 to −0.053), and burnout (β = −1.040, CI: −1.242 to −0.838).

**Conclusions:**

Nurses' job satisfaction was correlated with workplace bullying and burnout. Moreover, insufficient professional support from the authorities predicted nurses' job satisfaction. Reducing the instances of bullying and burnout among nurses, as well as improving their working environment, are essential to increase job satisfaction. This is possible with the support of hospital management, policymakers, and government authorities.

## 1 Introduction

Satisfaction is a complex and multifaceted factor that influences how people feel about activities, things, and other people [1]. Job satisfaction is a degree of affection or feeling for an individual's job and its primary components, and it is regarded as a positive notion that describes employee's working behaviors [2]. The aspects of having demands and wishing to achieve goals and commitment to the organization exist concurrently in terms of job satisfaction [3]. Human resources are critical components for enhancing the health care system's effectiveness. Achieving national and international health-related goals requires a sufficient number of skilled and motivated healthcare professionals as well as adequate financing and resources [4]. Numerous studies on nurse job satisfaction have been conducted globally; however, high levels of job dissatisfaction persist among nurses that were induced by a wide range of factors, including socio-demographic and workplace-related determinants [5,6]. In low-and middle-income countries, poor working conditions and a lack of resources are lowering nurses' job satisfaction and motivation, which may affect the standard of care and attrition rates.

Workplace bullying is a serious social issue that has been the topic of several studies, and nurses were more likely to report being bullied than other employees in the healthcare sector [7,8]. Continuous exposure to stressful events resulting from workplace bullying is linked to an increased risk of hypertension and cardiovascular disease [9], as well as mental health difficulties such as depression, anxiety, and posttraumatic stress disorder that can even lead to suicide [[10], [11], [12]]. Furthermore, several pieces of research demonstrated that bullying in the workplace can lead to a decrease in job satisfaction and an increase in burnout [13,14].

Burnout is a state of emotional fatigue and depersonalization and often a decrease in personal accomplishments, which results in unmanaged work-related stress [15]. There is a multitude of factors that can lead to burnout in nurses, including working night shifts, job-related stress, having a limited number of days off, having conflicts with other employees or patients, and the quality of the relationship between the nurse and their supervisor [[16], [17], [18], [19]]. In the long run, burnout has a negative effect on job satisfaction, which lowers the quality of care. Researchers found that nurses’ burnout ranged from 10% to 78% in 1,105 general acute care hospitals across Europe and the US, while job dissatisfaction ranged from 11% to 56% [20].

The shortage of nurses is a recognized concern worldwide, whereas Bangladesh has an estimated shortage of 280,000 nurses [21], making the country one of the 57 countries with a critical workforce shortage [22]. Job satisfaction is the most essential component, providing significant evidence for the notion that turnover intention was anticipated [23]. Moreover, the overwhelming COVID-19 outbreak triggered a wave of bullying and violence toward healthcare professionals [24]. A study carried out in Bangladesh during COVID-19 found that nurses exposed to workplace violence had a considerably higher intention to leave their jobs than nurses who were not exposed to workplace violence [25]. Another study conducted in Bangladesh found that nurses who experienced any form of emotional or workplace abuse had a higher level of depression, anxiety, and stress [26]. Also, the nurses lost their friends and family members due to the COVID-19 infection [27]. These traumatic experiences have been found to raise stress levels and exacerbate the psychological consequences as a result of moral injuries [28]. Consequently, these stressful events and the high frequency of workdays affected nurses' job satisfaction, life satisfaction, and turnover intention [29]. Besides, Piotrowski et al. found that during COVID-19, nurses’ lower resilience was significantly associated with their lower job satisfaction [30]. Age, gender, educational level, work experience, working conditions, degree of training, use of personal protective equipment, socioeconomic status, social support, and organizational support influenced nurses' resilience during the COVID-19 pandemic [31,32]. Whenever nurses experience better levels of job satisfaction, their morale and dedication grow, making it more likely that they will remain in the profession [33]. Furthermore, a previous study found links between job satisfaction and adverse patient outcomes [34]. Thus, the nurses' optimum level of job satisfaction is considered crucial in providing high-quality service, improving the entire healthcare force, and preparing the team for any sudden health crisis.

However, the only small-scale study conducted in 2016 in a specialized hospital in Bangladesh found a moderate level of job satisfaction among nurses [35]. To yet, no substantial evidence of Bangladeshi nurses' job satisfaction level was found that addressed the wide range of factors that were linked with predicting their job satisfaction. As the relationship of workplace bullying and burnout with job satisfaction is still unexplored comprehensively among Bangladeshi nurses, it is essential to reveal the association of these factors with nurses’ job satisfaction, as well as to identify the associated factors. Therefore, the current study investigated the relationship of workplace bullying and burnout with job satisfaction, as well as identified the demographic and occupational factors associated with job satisfaction among Bangladeshi nurses.

## 2 Methods

### 2.1 Study design, settings, and population

This study was of a cross-sectional design, and it was carried out between February 26, 2021 and July 10, 2021, among Bangladeshi registered nurses who were available on various social media platforms and nurses who were employed in one of eight selected tertiary hospitals in the two largest administrative divisions, which were Dhaka and Sylhet. To become graduated as a nurse, a student must complete a diploma (3-year program), or a bachelor's (4-year program) degree in Bangladesh [36]. Nurses can achieve a higher level of education (master's or PhD) after completing their undergraduate degrees. However, the nurses would have to meet the following requirements to participate in this study: (1) be Bangladesh Nursing and Midwifery Council (BNMC) registered nurses, (2) work in clinical settings, (3) be willing to participate, and (4) have at least one year of experience. We did not include any nurses who were working in faculty positions in any institution or who were not working in any hospital/clinical settings.

### 2.2 Sample size calculation

There were no reliable statistics available from the past about the percentage of nurses in Bangladesh who were satisfied with their job. So, based on the assumption that 50% of nurses were satisfied with their job, with 80% power, 95% confidence interval of 0.05–1.96, and with a 3% margin of error, the required sample size was calculated at 1,054. However, we intended more samples to be included to minimize the margin of error. As a result, we included more samples during the data collection, and the final analysis included a total of 1,264 responses.

### 2.3 Questionnaire development

A semi-structured questionnaire was developed for data collection based on a rigorous literature review. The questionnaire included the demographic and occupational variables along with the measurement tools for workplace bullying, burnout, and job satisfaction. For content validity, two clinical nurses and two public health experts in Bangladesh reviewed the preliminary questionnaire and provided their comments. After addressing their comments, the final questionnaire was modified further. Moreover, to assess construct validity, the inter-items correlation of the measurement tools was checked. For checking the reliability of the measurement tools, the confirmatory factor analysis, McDonald's omega (ω) was calculated [37]. However, before starting the final questionnaire dissemination, it was piloted on 20 clinical nurses, and they were not considered in the final analysis.

### 2.4 Measurement tools

#### 2.4.1 Workplace bullying

The 9-item “Short Negative Acts Questionnaire (S-NAQ-9)” was used to measure workplace bullying exposure among nurses [38]. It consists of nine questions that determine whether an individual has been bullied in the previous six months. The items on the scale include both the personal and the work-related types of bullying (for example, “there has been gossip or rumors spread about you,” and “necessary information was withheld that impeded your ability to do your job”). The response options varied from 1 to 5, with 1 indicating “never” and 5 indicating “daily.” Thus, the scale's overall score extends from 9 to 45, where a higher score exhibiting higher bullying. This scale was used to assess bullying in several studies conducted in Belgium, Italy, and Norway [[39], [40], [41]]. In our investigation, the S-NAQ-9 had a ω (McDonald's omega) of 0.88, indicating a good internal consistency in the current sample.

#### 2.4.2 Burnout

The 10-item “Burnout Measure-Short version (BMS-10)” developed by Malach-Pines was utilized in this study to measure burnout [42]. The BMS-10 is a quick and easy tool to evaluate burnout. A participant's degrees of physical exhaustion, emotional exhaustion, and mental exhaustion are measured in a series of 10 questions using the fundamental characteristics of the thought of burnout. On a Likert scale of seven points, ranging from 1 (never) to 7 (always), each item was given a rating. Thus, the total response scores for all ten items ranged anywhere from 10 to 70, depending on the response value for each item. Each participant's total burnout score was computed by dividing the sum of their response values by 10. As a result, the cumulative burnout score ranged between 1 and 7. The BMS-10 was validated and utilized on a variety of samples, and its psychometric properties were found to be satisfactory [[43], [44], [45]]. The ω for the BMS-10 was 0.89 showing good reliability in our study.

#### 2.4.3 Job satisfaction

The 5-item Short Index of Job Satisfaction (SIJS-5) was used in this study to measure the nurses' job satisfaction [46,47]. It is a self-report psychometric tool created by Brayfield and Rothe. The scale items include the respondents' perspective toward the job that determines their job satisfaction level. Participants were asked to rate each item on a five-point scale, with 1 representing "strongly disagree" and 5 representing "strongly agree”. As a result, each participant's overall job satisfaction score ranged from 5 to 25, with no cut-off value; higher scores implied higher job satisfaction. This 5-item SIJS has been used and validated in an earlier study [48]. This tool was also used in the study conducted during the COVID-19 pandemic [43]. In this study, the ω was found to be 0.64, which indicates that the internal consistency of this scale is good.

### 2.5 Independent and dependent variables

The independent variables were demographic variables (i.e., sex, age, marital status, educational level, and monthly salary), occupational variables (i.e., type of job, level of hospital, administrative division of workplace, weekly working hours, working department, sufficient equipment, years of experience, and timely payment), workplace bullying, and burnout. The nurse's job satisfaction was the dependent variable of the current study.

### 2.6 Data collection and recruitment procedure

We used a non-random convenience sampling strategy in this study. Both online and offline strategies were considered for self-response data collection. On the questionnaire's front page, the aims of the study, objectives, and eligibility criteria were presented. We provided training to 20 undergraduate nursing students that we selected specifically for the purpose of data collection. For collection of data online, the questionnaire was transferred to "Google Form", and an online link was generated. The trained data collectors shared the questionnaire link on nurses' social media platforms. These platforms included Facebook, Messenger, and WhatsApp groups. When the nurses clicked on the link to access the questionnaire, they were asked for their online consent to take part in the study. Upon approval, they got access to the main part of the questionnaire. This electronic data collection technique yielded 721 samples. To ensure the required sample size, an additional 700 printed version of questionnaires were sent out to nurses working at eight different tertiary hospitals in Bangladesh. These hospitals were located in Dhaka and Sylhet, which are the two largest and important administrative divisions in the country. The respondents were given one week to fill out the questionnaire, and after one week had elapsed, the data collectors received the completed questionnaires from the respondents. Finally, data collectors received 655 hard copies of the questionnaires; 543 were obtained as completed. Thus, the completed responses in total were 1,264 in the current study. The whole recruitment process is presented in Fig. 1, which was published elsewhere in an article from the same project [49].

**Fig. 1:** Flowchart of the recruitment process.

### 2.7 Data analysis

Data were analyzed and managed using STATA 16 and Microsoft Excel 2016. An Excel spreadsheet was used to compile the results of the offline and online data collection methods. Then, the sheet was imported into STATA so that further analysis could be performed. For categorical variables, descriptive statistics i.e., percentages and frequencies were calculated, whereas, for continuous variables, the mean and standard deviation were calculated. Inferential statistics, such as the *t*-test and the one-way analysis of variance (ANOVA), were utilized to estimate the mean differences in job satisfaction levels across a variety of demographic and occupational characteristics. To investigate the correlation between age, job satisfaction, workplace bullying, and burnout, the Pearson's correlation test was performed. Multiple linear regression models were fitted to investigate the adjusted association. The demographic and occupational factors associated with job satisfaction at a priori specified p-value of 0.1 in the *t*-test or ANOVA test, and age, sex, bullying, and burnout were included in subsequent multiple linear regression analyses to identify significant predictors for job satisfaction. We fitted three models for the adjusted association. In Model 1, demographic variables were included. In Model 2, occupational variables were included along with demographic variables. Model 3 included workplace bullying and burnout along with both demographic and occupational variables. Finally, multiple hierarchical regression models were performed to explore the contributory role of the study variables. A post-estimation test VIF was performed to determine the multi-collinearity. In this current study, p < 0.05 was considered statistically significant.

### 2.8 Ethics

Participation in this study was entirely voluntary. Participants provided their informed consent after understanding the study's goals and objectives. In this study, the “Helsinki Declaration 2013” guideline was adhered [50]. The “Begum Rabeya Khatun Chowdhury Nursing College's ethics committee” in Sylhet, Bangladesh, gave their official approval to conduct this study (Reference ID: BRKCNC/IRB/2021/5).

## 3 Results

### 3.1 Demographic and occupational characteristics of the participants

Table 1 presents the demographic and occupational characteristics of the participants**.** Most of the nurses were female (70.02%), and the mean age was 28.41 (±5.54) years. Over half of the participants were married (53.40%), and most had a diploma degree (41.14%). More than two-thirds of the participants (71%) had a monthly income above 21,000 BDT. The majority of the nurses worked in government (59.81%) and tertiary (71.99%) level hospitals primarily based in Dhaka (48.89%). The highest number of responses came from the critical ward (25.32%) and the medicine ward (25.79%). An almost equal number of nurses had an experience of <3 years (34.41%), 3–5 years (31.96%), and ≥6 years (33.62%). Over half of the nurses responded that they had to work with inadequate equipment (52.93%), and 10.28% of nurses did not receive their salary on time.

**Table 1:** Demographic and occupational characteristics of participants (n = 1,264).

Demographic variables	n	Percent/Mean (SD)
**Sex**		
Male	379	29.98
Female	885	70.02
**Mean age (year)**		28.41 (5.54)
**Age group (year)**		
<25	303	23.97
25-29	604	47.78
≥30	357	28.24
**Marital status**		
Unmarried	589	46.60
Married	675	53.40
**Educational level**		
Diploma degree	520	41.14
Bachelor's degree	514	40.66
Master's degree or above	230	18.20
**Monthly salary**		
<21,000 BDT	361	28.86
21,000–29,999 BDT	513	41.01
≥30,000 BDT	377	30.14
**Occupational variables**	**n**	**Percent**
**Type of job**		
Government	756	59.81
Private	508	40.19
**Level of hospital**		
Primary	147	11.63
Secondary	207	16.38
Tertiary	910	71.99
**Administrative division of workplace**		
Dhaka	618	48.89
Chattogram	132	10.44
Sylhet	375	29.67
Others^a^	139	11.00
**Work department**		
Critical ward	320	25.32
Emergency	80	6.33
General ward	197	15.59
Gynecological ward	97	7.67
Medicine ward	326	25.79
Surgery ward	244	19.30
**Weekly working hours**		
≤ 36 h	597	47.34
37–48 h	520	41.24
>48 h	144	11.42
**Years of experience**		
<3 years	435	34.41
3–5 years	404	31.96
≥6 years	425	33.62
**Sufficient equipment to manage patients**		
Yes	595	47.07
No	669	52.93
**Timely salary**		
Yes	1,134	89.72
No	130	10.28
**Workplace bullying (mean score)**		17.64 (7.29)
**Burnout (mean score)**		3.00 (1.21)
**Job satisfaction (mean score)**		17.30 (3.95)

SD = Standard Deviation; n = Number.

a Others = Rajshahi, Khulna, Barishal, Rangpur, Mymensingh.

The mean scores for workplace bullying, burnout, and job satisfaction were 17.64 (±7.29), 3.00 (±1.21), and 17.30 (±3.95), respectively.

### 3.2 Job satisfaction according to demographic and occupational characteristics

The mean differences in job satisfaction scores in different demographic and occupational characteristics are presented in Table 2. The married nurses had a significantly higher job satisfaction score (17.59 ± 4.02) than unmarried nurses (p = 0.006). Similarly, nurses with diploma degrees (17.71 ± 3.92), having 21,000 to 29,999 BDT monthly salary (17.68 ± 3.94), nurses from Chattogram division (18.16 ± 4.29), working as government employees (17.65 ± 3.90), working in the gynecological ward (17.89 ± 4.18), having sufficient equipment to manage patients (17.82 ± 3.95), and receiving a timely salary (17.51 ± 3.92) had significantly higher job-satisfaction scores compared to other groups within the same category (p < 0.05).

**Table 2:** Job satisfaction according to demographic and occupational characteristics.

Demographic variables	Job Satisfaction		
	Mean ± SD	F/t value	p value
**Sex**			
Male	17.20 ± 3.85	−0.58	0.561
Female	17.35 ± 3.99		
**Age group (year)**			
<25	16.96 ± 3.85	1.91	0.149
25-29	17.32 ± 4.09		
≥30	17.57 ± 3.78		
**Marital status**			
Unmarried	16.97 ± 3.84	2.78	0.006
Married	17.59 ± 4.02		
**Educational level**			
Diploma degree	17.71 ± 3.92	5.34	0.005
Bachelor's degree	16.91 ± 3.82		
Master's degree or above	17.26 ± 4.21		
**Monthly salary**			
<21,000 BDT	16.45 ± 3.87	11.91	<0.001
21,000–29,999 BDT	17.68 ± 3.94		
≥30,000 BDT	17.60 ± 3.94		
**Occupational variables**			
**Type of job**			
Government	17.65 ± 3.90	3.87	<0.001
Private	16.78 ± 3.96		
**Level of hospital**			
Primary	17.84 ± 4.38	1.85	0.158
Secondary	17.42 ± 4.03		
Tertiary	17.19 ± 3.85		
**Administrative division of workplace**			
Dhaka	17.08 ± 3.89	4.82	0.002
Chattogram	18.16 ± 4.29		
Sylhet	17.08 ± 3.81		
Others^a^	18.06 ± 4.06		
**Work department**			
Critical ward	17.48 ± 3.85	2.34	0.04
Emergency	17.08 ± 3.37		
General ward	17.35 ± 4.46		
Gynecological ward	17.89 ± 4.18		
Medicine ward	17.51 ± 4.00		
Surgery ward	16.60 ± 3.57		
**Weekly working hours**			
≤ 36 h	17.13 ± 3.71	1.54	0.214
37–48 h	17.53 ± 4.14		
>48 h	17.13 ± 4.17		
**Years of experience**			
<3 years	17.06 ± 3.87	2.21	0.111
3–5 years	17.23 ± 4.18		
≥6 years	17.62 ± 3.78		
**Sufficient equipment to manage patients**			
Yes	17.82 ± 3.95	4.41	<0.001
No	16.84 ± 3.89		
**Timely salary**			
Yes	17.51 ± 3.92	5.54	<0.001
No	15.51 ± 3.70		

SD = Standard Deviation; n = Number.

a Others = Rajshahi, Khulna, Barishal, Rangpur, Mymensingh.

### 3.3 Pearson's correlations among age, workplace bullying, burnout, and job satisfaction

Table 3 presents Pearson's correlations among age, workplace bullying, burnout, and job satisfaction. The correlation matrix reveals that workplace bullying, and job satisfaction were significantly positively correlated with respondents' age (p < 0.01). On the other hand, workplace bullying, as well as burnout, was found to have a significant negative correlation with job satisfaction (p < 0.001). Moreover, workplace bullying was found to have a significant positive correlation with burnout (p < 0.001).

**Table 3:** Pearson's correlations among respondents' age, workplace bullying, burnout, and job satisfaction.

Variables	1	2	3	4
1. Age	1			
2. Workplace bullying	0.124***	1		
3. Burnout	0.007	0.570***	1	
4. Job satisfaction	0.073**	−0.340***	−0.425***	1

**p < 0.01, ***p < 0.001.

### 3.4 Factors associated with job satisfaction

The results of three multiple linear regression models are presented in Table 4, which shows the associations between job satisfaction and other issues such as workplace bullying, burnout, demographic, and occupational factors. Only demographic variables were considered in **Model 1**. Compared to the nurses holding master's degrees or above, the diploma degree holders had higher job satisfaction (β = 0.916, CI: 0.268 to 1.564, p = 0.006). The respondents who were paid with monthly salary BDT 21,000–29,999 (β = 1.341, CI: 0.731 to 1.950, p < 0.001) and BDT ≥30,000 (β = 1.309, CI: 0.599 to 2.019, p < 0.001) had higher job satisfaction than the respondents who were paid with monthly salary BDT <21,000.

**Table 4:** Factors associated with job satisfaction identified from multiple linear regression models.

Variables	Model 1		Model 2		Model 3	
	Coefficient, β (95% CI)	p value	Coefficient, β (95% CI)	p value	Coefficient, β (95% CI)	p value
**Sex**						
Male	Reference		Reference		Reference	
Female	−0.041 (−0.523 to 0.442)	0.868	−0.273 (−0.766 to 0.219)	0.277	0.199 (−0.257 to 0.656)	0.392
**Age group (year)**						
<25	Reference		Reference		Reference	
25-29	−0.100 (−0.736 to 0.535)	0.757	−0.076 (−0.714 to 0.562)	0.815	−0.177 (−0.756 to 0.401)	0.548
≥30	−0.188 (−1.011 to 0.635)	0.654	−0.176 (−1.040 to 0.688)	0.690	−0.082 (−0.867 to 0.703)	0.838
**Marital status**						
Married	Reference		Reference		Reference	
Unmarried	−0.431 (−0.938 to 0.077)	0.096	−0.452 (−0.952 to 0.048)	0.076	−0.445 (−0.901 to 0.011)	0.056
**Educational level**						
Master's degree or above	Reference		Reference		Reference	
Bachelor's degree	−0.081 (−0.700 to 0.538)	0.797	0.009 (−0.600 to 0.617)	0.978	−0.191 (−0.744 to 0.363)	0.499
Diploma degree	0.916 (0.268 to 1.564)	**0.006**	0.861 (0.224 to 1.498)	**0.008**	0.381 (−0.204 to 0.966)	0.202
**Monthly salary**						
<21,000 BDT	Reference		Reference		Reference	
21,000–29,999 BDT	1.341 (0.731 to 1.950)	**< 0.001**	0.731 (−0.038 to 1.499)	0.062	0.660 (−0.036 to 1.355)	0.063
≥30,000 BDT	1.309 (0.599 to 2.019)	**< 0.001**	0.722 (−0.093 to 1.537)	0.082	0.589 (−0.150 to 1.328)	0.118
**Type of job**						
Government			Reference		Reference	
Private			−0.901 (−1.640 to −0.162)	**0.017**	−0.777 (−1.447 to −0.107)	**0.023**
**Administrative division of workplace**						
Dhaka			Reference		Reference	
Chattogram			0.854 (0.099 to 1.609)	**0.027**	0.889 (0.205 to 1.572)	**0.011**
Sylhet			−0.057 (−0.570 to 0.457)	0.829	−0.333 (−0.804 to 0.138)	0.166
Others^a^			0.993 (0.273 to 1.713)	**0.007**	0.895 (0.243 to 1.547)	**0.007**
**Work department**						
General ward			Reference		Reference	
Critical ward			0.184 (−0.507 to 0.875)	0.601	0.420 (−0.208 to 1.049)	0.190
Emergency			−0.607 (−1.626 to 0.412)	0.243	−0.164 (−1.093 to 0.764)	0.729
Gynecological ward			0.654 (−0.282 to 1.591)	0.171	0.847 (−0.008 to 1.702)	0.052
Medicine ward			0.074 (−0.614 to 0.762)	0.833	0.162 (−0.465 to 0.789)	0.612
Surgery ward			−0.735 (−1.482 to 0.012)	0.054	−0.694 (−1.373 to 0.015)	0.045
**Sufficient equipment to manage patients**						
Yes			Reference		Reference	
No			−1.230 (−1.696 to −0.763)	**< 0.001**	−0.541 (−0.974 to −0.107)	**0.015**
**Timely salary**						
Yes			Reference		Reference	
No			−1.475 (−2.221 to −0.729)	**< 0.001**	−0.697 (−1.380 to −0.013)	**0.046**
**Workplace bullying**					−0.086 (−0.120 to −0.053)	**< 0.001**
**Burnout**					−1.040 (−1.242 to −0.838)	**< 0.001**

Model 1 included demographic variables.

Model 2 included demographic variables plus occupational variables.

Model 3 included demographic variables, occupational variables plus bullying and burnout.

a Others = Rajshahi, Khulna, Barishal, Rangpur, Mymensingh.

In **Model 2**, occupational variables were included along with demographic variables. The private-employed nurses were significantly predicted to have lower job satisfaction than government-employed nurses (β = −0.901, CI: −1.640 to −0.162, p = 0.017). Compared to the nurses in Dhaka, the capital of Bangladesh, the nurses in Chattogram (β = 0.854, CI: 0.099 to 1.609, p = 0.027) and the nurses in other divisions (β = 0.993, CI: 0.273 to 1.713, p = 0.007) likely to have higher job satisfaction. Nurses without sufficient equipment to manage patients (β = −1.230, CI: −1.696 to −0.763, p < 0.001), and nurses not paid with on time (β = −1.475, CI: −2.221 to −0.729, p < 0.001) predicted to have significantly lower job satisfaction.

Workplace bullying and burnout were included in **Model 3** along with other demographic and occupational variables. Nurses' job satisfaction levels were decreased with a higher degree of workplace bullying (β = −0.086, CI: −0.120 to −0.053, p < 0.001). Similarly, nurses’ job satisfaction level was reduced when the nurses had a higher level of burnout (β = −1.040, CI: −1.242 to −0.838, p < 0.001).

### 3.5 Predicting factors of job satisfaction

The hierarchical linear regression models to predict job satisfaction is presented in Table 5. Our initial model in **Block 1** (demographic variables) explains 2.3% of the variance in job satisfaction scores. The addition of occupational variables in **Block 2** explained a 5% additional variance in the job satisfaction score. Finally, the inclusion of workplace bullying and burnout in **Block 3** contributed to explaining the 16.2% additional variance in job satisfaction scores beyond the previous models. All of these increments were statistically significant (p < 0.001).

**Table 5:** Predicting factors of job satisfaction.

Variables	Block 1 (β)	Block 2 (β)	Block 3 (β)
Sex	−0.026	−0.147	0.290
Age (year)	−0.044	−0.260	−0.240
Marital status	−0.422	−.439	−0.459
Educational level	0.519**	0.486**	0.250
Monthly salary	0.612**	0.375	0.350*
Type of job		−1.140***	−0.998**
Administrative division of workplace		0.194	0.123
Work department		−0.119	−0.136*
Sufficient equipment to manage patients		−1.257***	−0.580**
Timely salary		−1.388***	−0.594
Workplace bullying			−0.084***
Burnout			−1.028***
F	5.725***	9.599***	30.953***
R^2^	0.023	0.072	0.234
ΔR^2^	0.023***	0.050***	0.162***

*p < 0.05, **p < 0.01, ***p < 0.001.

## 4 Discussion

Nursing as a profession plays an essential role in ensuring safety and elevating the suffering of patients since nurses provide immediate care and spend the vast majority of their work time with them. A healthy working environment is related to high-quality care and lower adverse patients' health consequences. Liu et al. (2019) emphasized that unsafe and intimidating workplaces were associated with job dissatisfaction among healthcare workers [51]. Our study explored the association of workplace bullying and burnout with nurses’ job satisfaction and addressed the associated demographic and occupational factors. Clinical nurses from different geographical parts of Bangladesh participated in this study.

This study found that workplace bullying, and burnout were significantly correlated with nurses' job satisfaction. While workplace bullying and burnout increased, nurses' job satisfaction significantly decreased. Our findings were supported by several previously conducted studies in many countries that found that nurses were at greater risk of assault and abusive language than physicians were, and bullying and harassment were crucial factors affecting nurses' job satisfaction [[52], [53], [54]]. Furthermore, Pérez-Fuentes et al. (2020) found that internally and externally, nurses' job satisfaction was negatively impacted by aggression and bullying by colleagues, patients’ relatives, and other people accompanying the patient [55]. After the COVID-19 pandemic, many incidences of stigmatization, violence, and harassment against patients, healthcare employees, and medical infrastructures were reported, with 67% targeting healthcare workers [24]. Moreover, frontline nurses had significant challenges in terms of their mental health during the COVID-19 pandemic [26]. Pandemics pose a significant threat to healthcare professionals in Bangladesh, because many of its hospitals and clinics have limited resources [56]. A lack of employee welfare programs and support from the authorities at the workplace during the COVID-19 pandemic was also observed in Bangladesh, which might influence nurses' satisfaction levels with their job [57].

This study found that nurses' demographic and occupational characteristics were significantly associated with job satisfaction. Diploma degree holders had higher job satisfaction than master's degree holders. A study found that educational qualification and level were important factors in job satisfaction [58]. However, in our research, nurses with lower academic degrees exerted higher level of job satisfaction. This may be due to the fact that the salary grade and promotional system are almost similar for all nurses throughout the level of education, and the nursing profession in Bangladesh is considered to be of lower social standing, get lower financial pay, and hold a lower status at work than other professions [59]. Our findings can also be explained by the previous research that nurses with higher levels of education continue to have a higher risk of psychological suppression when taking into consideration the social impression, the low wage increments, and the lack of professional advancement that are available in Bangladesh [26], which ultimately impact their job satisfaction level. We found that nurses serving in the private sector were less satisfied than those who were serving in the government sector. A recent study conducted in Bangladesh during COVID-19 reported that privately employed nurses were more likely to leave their job than publicly employed nurses [25]. The possible reason could be the lack of personal protective equipment and the support from the respective authorities [60]. Moreover, during COVID-19, the ministry of health in Bangladesh disbursed the incentives only to government employees [61]. Our finding was also supported by a study conducted in Bangladesh, which indicated that nurses working in specialized public hospitals were more satisfied, and their satisfaction was associated with organizational dedication and top management support [35]. This finding may also be explained by nurses' monthly salary and their timely payments. Our research revealed that nurses who were paid high salaries and paid on time were more satisfied with their job. In Bangladesh, nurses in the government sector are paid high wages, and they are also paid on time. Jackson and Schuler (2006) reported that timely salary affects attracting good employees and maintaining performance, and it is becoming increasingly crucial in the highly challenging global economy [62]. Moreover, findings from study showed that prioritizing timely payments helped attract and retain the best and brightest workers and enhance their job satisfaction [63]. This study identified workplace areas as a significant predictor of nurses' job satisfaction. Nurses working in Chattogram or other divisions were more satisfied with their job than nurses working in Dhaka, the busiest city and the capital of Bangladesh. It is a fact that nurses in Dhaka have to deal with a large number of patients with limited resources. A previous study demonstrated that long working hours and staff shortages were the main reasons for dissatisfaction in the busiest hospitals, and thus, the staff feels less secure, which may lessen their job satisfaction [64].

Our research found that nurses were satisfied at work while they had enough supplies of needed equipment. Similarly, several investigations reported a positive association between the supply of required equipment and job satisfaction [65,66]. Furthermore, Yu et al. (2018) described that individuals reported having more positive views on their jobs when their total requirements were met, which suggests that the supply of needs is associated with job satisfaction [67]. When people observe a perfect match between their requirements and a supply that satisfies their task, they deduce meaning and significance from the fact that they are acknowledged as desired and necessary. For instance, Basit et al. (2016) reported that psychological safety was promoted by the fit of a need-supplies, which indicates that workers believe their workplace is more favorable for participation than their identity, reputation, and career progression has not been jeopardized [68].

We believe that our study findings can assist the corresponding authorities in taking corrective action and ensuring a possibly safer working environment for the nurses to enhance their job satisfaction.

### 4.1 Strengths and limitations

This is the first study of its kind to investigate the relationship of job satisfaction with bullying and burnout in the workplace among Bangladeshi registered nurses. The measurements of three important job-related issues in a single study provided a more significant opportunity to analyze the relationship between these concerns. By sending out invitations to nurses in every part of the country, we were able to obtain a representative and optimal sample size. Nevertheless, this study was not without its limitations. Avoiding selection bias was not possible because of using a non-random sampling technique. Due to the fact that the data were collected through self-reporting questionnaires, there was the possibility of information bias. Due to a cross-sectional design, causality could not be determined. Finally, it was not possible to evaluate the direct influence of COVID-19 on nurses' job satisfaction because there were no data available prior to COVID-19. Therefore, we suggest further studies with large sample size utilizing a random approach and focusing on a wide variety of factors, including workplace environment and safety issues that are related to the nurses’ job satisfaction.

## 5 Conclusions

Bangladeshi nurses' job satisfaction was significantly associated with workplace bullying and burnout. Job types, geographical location of the workplace, sufficient equipment supplies, and timely payment significantly predicted the nurses' job satisfaction. Therefore, the respective authorities’ insufficient professional support is assumed to exist at the workplace, which might hinder nurses' level of job satisfaction. In order to increase job satisfaction, it is necessary for hospital management, policymakers, and the government authorities to support and implement suitable policies to address the factors, promote the working environment for nurses, and reduce the incidence of burnout and bullying in the workplace. There is a need for additional rigorous research on similar issues in order to create safe and sustainable work environments.

## Author contribution statement

Saifur Rahman Chowdhury; Humayun Kabir: Conceived and designed the experiments; Performed the experiments; Analyzed and interpreted the data; Contributed reagents, materials, analysis tools or data; Wrote the paper.

Nahida Akter; Mohammad Azmain Iktidar; Mahfuzur Rahman Chowdhury; Ahmed Hossain: Contributed reagents, materials, analysis tools or data; Wrote the paper.

## Funding statement

This research did not receive any specific grant from funding agencies in the public, commercial, or not-for-profit sectors.

## Data availability statement

Data will be made available on request.

## Declaration of interest's statement

The authors declare no conflict of interest.
